The article "Cytokine Changes in the Aqueous Humor in Rubella-Related Fuchs Heterochromic Iridocyclitis" was published in 2022. Journal: Dis Markers.

# Cytokine Changes in the Aqueous Humor in Rubella-Related Fuchs Heterochromic Iridocyclitis

**DOI:** 10.1155/2022/8906752

**Published:** 2022-02-07

**Authors:** Yi Mao, Sijie Lin, Chengfang Zhu, Xiaodong Liu, Huping Wu, Shangkun Ou

**Affiliations:** ^1^Eye Institute and Affiliated Xiamen Eye Center of Xiamen University, School of Medicine, Xiamen University, Xiamen, Fujian 361002, China; ^2^Fujian Key Laboratory of Ocular Surface and Corneal Diseases, Xiamen University, Xiamen 361002, China

## Abstract

This retrospective study is aimed at determining the correlation between cytokine levels and virus status in the aqueous humor of 38 patients with Fuchs heterochromic iridocyclitis (FHI) with/without a viral presence between May 2017 and January 2020. The levels of cytokines were analyzed in the groups with and without virus-related FHI. Among the patients, 50% had rubella virus, 5.26% had cytomegalovirus, and 2.63% had herpes simplex virus infections. The expression of interleukin-6 (IL-6) and IL-8 was significantly higher, and that of basic fibroblast growth factor (bFGF) was significantly lower in the virus-positive group than in the virus-negative group (*P* = 0.015, *P* = 0.001, and *P* = 0.001, respectively). Although there was no significant difference in the mean expression of vascular cell adhesion protein 1 (VCAM-1), IL-10, and vascular endothelial growth factor (VEGF), that of VCAM-1 and IL-10 was higher (*M* = 1338 and *M* = 1390, respectively; *M* = 6.225 and 10.600, respectively) and that of VEGF was lower (*M* = 134.5 and *M* = 38.70, respectively) in the virus-positive group than in the virus-negative group. Similar findings were observed for the expressions of IL-6, IL-8, and bFGF in the rubella-positive and rubella-negative groups. Viral presence was highly related to FHI, especially that of the rubella virus. High levels of inflammatory cytokines and low levels of neovascularization-related factors are involved in rubella-related FHI. These study findings could be helpful in the diagnosis and treatment of FHI.

## 1. Introduction

Fuchs heterochromic iridocyclitis (FHI) is a chronic, usually unilateral, nongranulomatous uveitis of insidious onset. It is characterized by iris depigmentation, accounting for approximately 0.5–7% of all cases with uveitis [1–3]. However, FHI is commonly misdiagnosed because of its easily neglected and diverse manifestations [4]. The typical characteristics of FHI are keratic precipitates (KPs), iris atrophy, nonpersistent inflammatory manifestations, vitreous infiltration, lens opacification, and secondary glaucoma with symptoms such as blurred vision [4]. Medium- or star-shaped KPs could be distributed in the cornea of the triangle area, pupil area, or diffusely posterior in patients with FHI. Ocular examination can also show light anterior chamber flare, a small number of aqueous cells, iris depigmentation, or iris atrophy. FHI patients are prone to have Koeppe nodules, posterior capsule opacification, ocular hypertension, opacity, and cells in the anterior vitreous. In addition, clinical manifestations such as abnormal corneal spots or corneal endothelium, abnormal blood–humor barrier, and nonpersistent inflammation can be found in FHI [5–11].

The article "Cytokine Changes in the Aqueous Humor in Rubella-Related Fuchs Heterochromic Iridocyclitis" was published in 2022. Journal: Dis Markers.

At present, the complex and varied symptoms of FHI make it difficult to diagnose. Misdiagnosis can result in unnecessary corticosteroid treatment or misinformed expectations about the progress of the condition. Many risk factors for FHI, including inflammation, tumor, trauma, surgery, congenital syndromes, nerve dysfunction, autoimmunity, and infection, have been studied [12]. However, viral pathogens are more regarded as potential causes of FHI; these include the herpes simplex virus (HSV and VZV) [13], cytomegalovirus (CMV) [14, 15], and rubella [16–18]. The predominant mechanisms involved in viral anterior uveitis are chronic inflammatory processes, [19] which are accompanied by changes in cytokine levels [20] and immunopathology [21].

Rubella virus infection highly correlates with FHI [16–18], with 68% of FHI patients infected with the rubella virus [22]. Rubella virus, a member of the *Riboviriad* family, *Matonaviridae* [23, 24], is the etiologic agent of rubella, which can induce congenital birth defects, miscarriage, and stillbirth via transplacental transmission [24–26]. Rubella occurs worldwide during epidemics [27]. Although the global incidence of rubella has decreased with the development of vaccines, the number of congenital rubella syndrome cases is approximately 100,000 every year [28]. Rubella virus can persistently infect the eye for years [17].

In the eyes of those with Fuchs' uveitis syndrome, significantly higher levels of inflammatory factors (IL-6, IL-8, and IL-10) than those in senile cataract-affected eyes were detected because immune mediators are crucial to specific viral intraocular inflammation [22]. IL-6 and IL-8 have the potential to act as markers of inflammation in the aqueous humor in FHI.

The role of the intraocular presence of rubella during the development of FHI is controversial [18, 29] and the mechanism of rubella infection in FHI is not clear. In this study, we aimed to investigate the viruses involved in FHI, such as CMV, HSV, VZV, and rubella, and determine the correlation between cytokine levels and virus status in the aqueous humor of patients with FHI, especially in the case of rubella.

The article "Cytokine Changes in the Aqueous Humor in Rubella-Related Fuchs Heterochromic Iridocyclitis" was published in 2022. Journal: Dis Markers.

## 2. Materials and Methods

### 2.1. Study Design and Participants

The clinical data of 38 patients with FHI treated at the Xiamen Ophthalmology Hospital affiliated with Xiamen University between May 2017 and January 2020 were retrospectively analyzed. Ethical approval was obtained from the Institutional Review Board of Xiamen Ophthalmology Hospital affiliated with Xiamen University. The study procedures were performed in accordance with the principles of the Declaration of Helsinki. The diagnosis of FHI was based on the Standardization of Uveitis Nomenclature (SUN) classification criteria [30]: (1) heterochromia or unilateral diffuse iris atrophy; (2) characteristic KPs, anterior chamber cells, or anterior chamber inflammation; (3) unilateral uveitis; (4) no evidence of active retinitis; and (5) neither endotheliitis nor nodular, coin-shaped endothelial cell. Informed consent was obtained from patients or their guardians with FHI before collecting aqueous humor samples. A tenth of a milliliter of the aqueous humor was aspirated using a 30-gauge needle via limbal paracentesis after local anesthesia using the proparacaine hydrochloride eyedrop (ALCAINE 5 mg/mL, Alcon, USA).  Table 1 summarizes the demographic characteristics of the patients.

### 2.2. Aqueous Humor Virus Detection

The method has been described previously [29]. Briefly, the presence of rubella virus, CMV, HSV, and VZV in the aqueous humor was confirmed using an ELISA microplate reader (Biotek ELx 800). For viral quantification in samples, a software program was used to generate a four-parameter sigmoidal curve. The levels of CMV-IgG > 9 U/mL, HSV-IgG > 9 U/mL, HZV-IgG > 16 U/mL, and rubella-IgG > 10 U/mL indicated a positive result.

### 2.3. Assessment of Aqueous Humor Cytokine Levels

Flow cytometry was used to analyze the expression of vascular endothelial growth factor (VEGF), basic fibroblast growth factor (bFGF), IL-6, IL-8, IL-10, and vascular cell adhesion protein 1 (VCAM-1) using the BD CBA Human Soluble Protein Master Buffer Kit (BD, 558264). Results were analyzed using the FCAP Array™ software program.

### 2.4. Statistical Analysis

The parameters were compared using the Mann–Whitney *U* test between the FHI groups with and without viral infection. Continuous variables are presented as mean (*M*) and standard error of the mean for normally distributed variables and as median value and interquartile range for variables with skewed distribution. SPSS Statistics (version 22.0) was used to perform statistical analyses, and the threshold for statistical significance was set at *P* < 0.05.

## 3. Results

Aqueous humor specimens were collected from 38 patients whose conditions were diagnosed as FHI based on the SUN classification criteria; the patients had no other eye or systemic diseases. Twenty-four patients (63.16%) were women, and 14 (36.84%) were men. The mean age was 38 years (range, 14–69 years). The left and right eyes each accounted for 50% (*n* = 19) of the cases. The demographics and clinical information of patients with FHI are shown in Table 1.

The article "Cytokine Changes in the Aqueous Humor in Rubella-Related Fuchs Heterochromic Iridocyclitis" was published in 2022. Journal: Dis Markers.

Test results of the presence of intraocular viruses and antibody values of rubella virus, CMV, HSV, and VZV in the aqueous humor are shown in Table 2. Among 38 patients, 16 (42.11%) tested negative and 22 (57.89%) tested positive for the virus; 50% (*n* = 19) of the patients tested rubella positive, 5.26% (*n* = 2) tested CMV positive, 2.63% (*n* = 1) tested HSV positive, and none tested VZV positive. The presence of intraocular rubella virus infection was confirmed, consistent with the fact that most FHI patients were seropositive for this entity.

We divided the 11 patients who underwent measurements of the expression of cytokine levels in the aqueous humor into two groups (Table 3). The positive group (*n* = 5) had higher levels of IL-6 (*M* 145.767, SD 57.988) and IL-8 (*M* 185.100, SD 15.839) than the negative group (*n* = 7) (*M* 41.375, SD 8.432 and *M* 30.333, SD 9.616, respectively). The expression levels of VEGF, IL-10, and VCAM did not differ significantly between the two groups. However, the virus-positive group had a lower bFGF level (*M* 1.1, SD 0.17) than the virus-negative group (*M* 27.325, SD 6.749). Furthermore, we focused on cytokine changes in the aqueous humor of rubella-involved FHI patients, considering that half of the FHI patients had high intraocular antibody levels against rubella. IL-6 and IL-8 levels were significantly higher in the positive group than in the negative group (Figure 1). The bFGF expression was downregulated in the rubella-positive group, similar to that observed in the virus-positive group.

## 4. Discussion

FHI is a unilateral chronic nongranulomatous uveitis that is difficult to diagnose based on clinical manifestations alone, especially in the Chinese population. This is because these people generally do not have a different iris color of two eyes when iris depigmentation occurs owing to high pigment concentration, resulting in additional differential diagnoses. FHI is generally not detected until it causes secondary affection with late symptoms such as blurred vision and dark shadows that affect vision. In this study, we discovered the changes in inflammatory cytokines and virus antibody expression levels in aqueous humor specimens to yield strong evidence for FHI diagnosis.

HSV, VZV, and CMV are the predominant pathogens in a chronic inflammatory process with the involvement of viral anterior uveitis. However, less than 8% of patients with FHI tended to have an increased level of viral antibody expression (Table 1). Recent studies showed that rubella virus infection is a possible etiological agent of FHI [31]. This led us to hypothesize that active rubella virus infection is related to FHI, and the rubella antibody in the aqueous humor of these patients can help diagnose FHI. Rubella virus is associated with the pathogenesis of Fuchs' heterochromic uveitis, and nearly all European cases had active antibodies against the rubella virus in the aqueous humor [32]. The incidence of FHI has decreased after the introduction of vaccination against the rubella virus [31]. Several researchers have suggested that the presence of the rubella virus in the eye is not a prerequisite for the development of FHI. We carried out this study to ascertain the association between rubella virus infection and FHI by detecting the production of intraocular antibodies and to confirm the presence of the active rubella virus antibody in the aqueous humor of FHI patients.

The article "Cytokine Changes in the Aqueous Humor in Rubella-Related Fuchs Heterochromic Iridocyclitis" was published in 2022. Journal: Dis Markers.

Furthermore, we detected the levels of several proinflammatory cytokines, including IL-6, IL-8, IL-10, bFGF, VEGF, and VCAM, in the aqueous humor of FHI patients who underwent the examination. Immunoassays have been used to identify the distinct patterns of cytokines associated with both clinical disease and the cellular infiltrates present. First, VEGF, bFGF, and VCAM are all suggested as key regulators of vasculogenesis, and they can stimulate vascularization under inflammation in any type of disease. Reportedly, bFGF can improve leukocyte recruitment and endothelial cell adhesion molecule expression during inflammation [33]. In our study, we observed an obvious decrease in the level of bFGF in the aqueous humor in the virus-positive group compared with the virus-negative group, while there was no significant difference in VEGF or VCAM levels. There has been no relevant literature on the relationship between FHI and bFGF until now, as neovascularization in the iris in FHI cases has rarely been documented. The expression of bFGF in the aqueous humor could be a new observation index for FHI.

Bioinformatics plays a significant role in the pathogenesis of uveitis. There was a positive correlation between IL-6 and IL-8 levels and the number of neutrophils present in patients with uveitis aqueous humor associated with Fuchs' heterochromic cyclitis [34]. In our study, high concentrations of IL-6 and IL-8 were measured in the aqueous humor samples of patients with FHI, indicating that the anterior chambers of these patients had an increased number of neutrophils. A previous study found that the levels of IL-2, interferon-gamma, IL-10, and other cytokines are significantly higher in vitreous humor-derived T cells, and Fuchs' heterochromic cyclitis patients produce high levels of IL-10, which might help downregulate the inflammatory response, resulting in benign clinical outcomes [35]. However, two groups of patients with FHI having the same level of IL-10 suggested no significant difference in the accumulation of T cells in the aqueous humor. As expected, FHI patients with rubella had downregulated expressions of bFGF and upregulated expressions of IL-6 and IL-8, similar to that observed in the virus-positive group. If patients had high expression levels of IL-6 and IL-8 and negative results for bFGF in the aqueous humor, we would be more certain when diagnosing virus-related FHI on the basis of suggested symptoms.

The article "Cytokine Changes in the Aqueous Humor in Rubella-Related Fuchs Heterochromic Iridocyclitis" was published in 2022. Journal: Dis Markers.

The presence of the rubella virus in the aqueous humor stimulates inflammation in patients with FHI (classic FHI phenotype). With the detection of an increased level of proinflammatory cytokines and a decreased expression of bFGF preventing vasculogenesis and the local persistence of the rubella virus, we obtained a new direction in the investigation of the pathomechanism and development of a treatment against the etiology of FHI.

The presence of the virus was highly associated with the classic phenotype of FHI, especially that of the rubella virus. This presence constantly causes inflammatory stimulation in the aqueous humor, resulting in significantly increased levels of proinflammatory cytokines, such as IL-6 and IL-8, and low levels of neovascularization-related factors like bFGF. The persistence of viruses and inflammatory cytokine levels in the aqueous humor of patients with FHI could help investigate the pathomechanism of FHI and develop cause-specific treatments.

However, it is unclear whether the virus detected and isolated from aqueous humor in the FHI patient was from acute infection, reinfection, or reactivation of latent virus. Further investigations should include the isolation and characterization of rubella virus strains associated with FHI. What is more, the correlation of symptoms and the rubella-related FHI should be confirmed in the future.

## Figures and Tables

**Figure 1:** The cytokine changes of aqueous humor in rubella-related FHI. VEGF was high in rubella-related FHI than the virus negative group (a). BFGF was significantly lower in rubella-related FHI (b). The IL6 (c) and IL8 (d) were significantly higher in the positive group. Although there was no significance in the IL10 (e) and VCAM (f), they were higher in the positive group than the negative group (^∗^*P* < 0.05).

The article "Cytokine Changes in the Aqueous Humor in Rubella-Related Fuchs Heterochromic Iridocyclitis" was published in 2022. Journal: Dis Markers.

**Table 1:** Demographics and clinical characteristics of FHI patients.

Case	38	
	Female	24 (63.16%)
	Male	14 (36.84%)
Age (years), median (range)	38 (14-19)	
Eye number	38	
	Left eye	19 (50%)
	Right eye	19 (50%)

**Table 2:** The rate of virus involved FHI.

Case	38	
Negative	16 (42.11%)	
Positive	22 (57.89%)	
	Rubella	19 (50%)
	CMV	2 (5.26%)
	HSV	1 (2.63%)
	VZV	0 (0%)

CMV: cytomegalovirus; HSV: herpes simplex virus-1; VZV: herpes simplex virus-2.

**Table 3:** Cytokines levels in all measured aqueous humor.

Cytokines	Negative group (*n* = 7)	Positive group (*n* = 5)	*P* value
VEGF (pg/mL), median (Std)	34.500 (1.153)	38.700 (11.879)	0.200
bFGF (pg/mL), median (Std)	27.325 (6.749)	1.100 (0.173)	0.001^∗^
IL6 (pg/mL), median (Std)	41.375 (8.4318)	145.767 (57.988)	0.015^∗^
IL8 (pg/mL), median (Std)	30.333 (9.616)	185.100 (15.839)	0.001^∗^
IL10 (pg/mL), median (Std)	6.225 (2.968)	10.600 (3.536)	0.530
VCAM (pg/mL), median (Std)	1338.333 (369.656)	1390.133 (438.769)	0.268

^∗^ *P* < 0.05. VEGF: vascular endothelial growth factor; bFGF: basic fibroblast growth factor; IL: interleukin; VCAM: vascular cell adhesion molecule.

## Data Availability

The data used to support the findings of this study are included within the article.
